The article "The Customs Clearance Efficiency of Guangdong-Hong Kong Land Transportation Based on BP Neural Network Algorithm" was retracted in 2023. Reasons: signs of a paper mill; suspected computer-generated content; unreliable results or conclusions; concerns about the data.

# The Customs Clearance Efficiency of Guangdong-Hong Kong Land Transportation Based on BP Neural Network Algorithm

**DOI:** 10.1155/2022/9964795

**Published:** 2022-07-31

**Authors:** Linyu You

**Affiliations:** Guangzhou Huaxia Vocational College, Guangzhou, Guangdong 510900, China

## Abstract

With the continuous development of the economy, the trade volume of customs clearance by land transportation between Guangdong and Hong Kong is increasing, but there are many problems in customs clearance by land transportation between Guangdong and Hong Kong. Therefore, it is necessary to start with the logistics mode of land transportation between Guangdong and Hong Kong, reduce the cost of customs clearance by land transportation between Guangdong and Hong Kong, and increase the trade volume by land transportation between the two places. This paper systematically analyzes the present situation of customs clearance efficiency in China and introduces BPNN (BP neural network) algorithm to optimize customs clearance. The detailed idea and process of the algorithm are introduced, and the BPNN trained by the algorithm is applied to function approximation. The simulation results show that this scheme can not only improve the convergence speed of the algorithm in the training process but also the trained BPNN has strong adaptive and self-learning ability. Comparing the customs clearance efficiency before and after the improvement, the results show that the improved customs clearance efficiency is higher and can save a lot of time, thus verifying the effectiveness and applicability of the model-solving algorithm.

## 1. Introduction

After the reform and opening up, Guangdong took the lead in opening the door to trade with the outside world. Therefore, the volume of import and export customs clearance in Guangdong has been at the forefront of China. Hong Kong is one of the four famous free trade ports in the world. Hong Kong Airport is the busiest airport in the world, and its cargo volume ranks first in the world for many years. Hong Kong Port is a natural port in China and a shipping center in the Far East. Hong Kong has a unique geographical location and relatively loose import and export policies [1]. Shenzhen is one of the cities with the strongest scientific and technological innovation ability and the most active economy in Guangdong, Hong Kong, Macao, and Greater Bay Area urban agglomeration with dense industrial clusters. In order to make the export of goods more convenient, many companies usually choose to use freight forwarders in the way of customs clearance, but in this process, a complicated process is needed, which reduces the efficiency of customs clearance to a certain extent and has a certain impact on the development of foreign trade. Therefore, this paper analyzes the problems in customs clearance, puts forward reasonable measures, and strives to improve customs clearance efficiency [2].

International freight transport does not attach importance to customs clearance customers in Guangdong and Hong Kong and lacks good service awareness. In Guangdong Province, most of the international freight companies usually regard sea freight or air freight forwarding as their main business within their business scope. The land transportation price between Guangdong and Hong Kong varies according to the nature of the goods. The profit margin of each vehicle is 200∼1000 yuan, which is relatively low compared with international transportation. At the same time, in the process of customs declaration and freight transportation, there are some factors to varying degrees, which lead to low profits in the process of business operation and the impact of difficulties in the process of operation. Therefore, there is a phenomenon that the carrier is unwilling to accept orders, and there is a phenomenon of negative service in the process of work. There is a widespread phenomenon of misrepresentation of miscellaneous expenses. In the process of land transportation, after the owner of the transportation company declares to the transportation company responsible for transportation business, expenses that must be declared on the receipt occur, such as warehousing fee and transit fee. During the transportation of goods, the transportation company should have charged the customer in strict accordance with the invoice. However, in the process of transportation, there is information asymmetry in many aspects. In terms of overtime fee and waiting fee (150 yuan per hour if waiting for more than 2 hours). The failure to communicate effectively and timely in all aspects of transportation has led some transportation companies to falsely report the waiting time or service fee. This situation persists, and even these false costs exceed the freight costs.

## 2. Related Work

At present, the research on the innovation ability of the port logistics industry cluster is even less, and it is mostly concentrated in a single field such as logistics or port. In the existing industry, the port industry and the logistics industry are closely related. Its comprehensive innovation capability directly affects the overall development of the port logistics industry cluster. Therefore, it is necessary to carry out research on the innovation ability of the port logistics industry cluster. Land transportation between Guangdong and Hong Kong is an important means of logistics, which can not only improve transportation efficiency but also improve customs clearance efficiency, thus having a significant impact on foreign trade. Therefore, some scholars have analyzed a series of problems existing in the land transport clearance between Guangdong and Hong Kong, optimized the clearance links, and made efforts to improve the clearance efficiency. Some researchers have analyzed the mechanism of the innovation ability of the port logistics industry cluster. According to the questionnaire statistics, the evaluation index system of the port logistics industry cluster is obtained. On this basis, the innovation ability of the port logistics industry cluster is quantitatively evaluated by using BP neural network algorithm. Taking the evaluation of the Ningbo port logistics industry cluster as an empirical case, the application steps of the BP neural network algorithm and the evaluation results are explained. Customs is in a very important position in port logistics. If the customs clearance efficiency is high, the goods can quickly pass through the port node. In order to facilitate export, export enterprises usually choose to arrange the land transportation and customs clearance of their goods through freight forwarders. However, the customs clearance process of Guangdong-Hong Kong land transportation is complicated, and the participants in the customs clearance process often have interest conflicts due to various reasons, which reduces the efficiency of customs clearance of Guangdong-Hong Kong land transportation, increases the transportation cost, and further affects the development of foreign trade. Liu et al. [3] study and discuss the customs clearance process of imported goods in international air cargo terminals and construct a Petri net to analyze the goods, information, and people flow in the process of importing goods. Zhao et al. [4], considering the influence of new information and communication technology, modeled the discrete multimodal transport system and managed from the operational level by using the time Petri net framework [5] and studied configurable process models in logistics by applying cases. It analyzes and creates a model of the import and export customs clearance service process [6] and processes and provides configurable process models from these models. Jiang et al. [7] make a comprehensive diagnosis and analysis of the department settings and functions and redesign the business process system according to the analysis results. Li [8] focuses on the analysis and research of several subsystems in the customs clearance process in order to find out the disadvantages existing in the current customs clearance process [9] and reorganize and improve the existing customs clearance management mode through process optimization and institutional arrangement by using the theory of risk management. Li e al. [10] set the modeling tools of customs clearance process reengineering as extended event process chain, generalized stochastic Petri net, and queuing Petri net. With the help of the analysis matrix of the extended event process chain, a customs clearance process reengineering scheme based on classified clearance is finally proposed. Shi and Zhao [11] study regional economic division and point out that on the whole, regional economic division reduces the efficiency of resource allocation and the total social output. In the longer term, the regional economic division has a very negative impact on the development of backward areas.

Customs clearance cycle, customs clearance efficiency, and customs clearance service quality have a significant impact on the import and export of goods of all enterprises and also indirectly affect the national economy [12]. The construction of a smooth customs clearance environment largely depends on the government's policy guidance and the coordination of various departments and links at the port. In the construction of port areas, bonded areas, and logistics parks, it is necessary for Guangdong-Hong Kong land transportation to “explore boldly, try first, and play a role” and explore new development modes under the guidance of government policies at all levels. Therefore, the customs clearance efficiency of goods in port logistics is increasingly concerned by multinational companies and logistics enterprises and has become the most direct factor affecting the trade and investment environment of a country or region. This paper analyzes the background of customs clearance efficiency and the factors restricting customs clearance efficiency. By using modern scientific means such as BPNN (BP neural network) algorithm and computer simulation technology, this paper analyzes the shortcomings in China's customs clearance process and puts forward optimization methods for China's customs clearance process with a view to improving the efficiency and business ability of Guangdong-Hong Kong land transportation clearance process.

## 3. Research Method

### 3.1. Mathematical Description of BPNN Algorithm

BPNN is one of the most widely used artificial neural networks, and its learning is divided into two parts: forward propagation and backward propagation [13, 14]. Its main principle is to train the input sample data and constantly modify the network connection weights and other parameters to make the error function decrease along the negative gradient direction so as to approach the expected output.

Because of its strong nonlinear mapping ability and self-learning ability, it has made outstanding achievements in many fields such as model identification and classification, time series prediction, and data mining. The network structure is shown in Figure 1.

Generally, the BPNN structure is composed of IL (input layer), HL (hidden layer), and OL (output layer). The number of neurons in IL corresponds to the number of input parameters in the network, and the number of neurons in OL corresponds to the number of output values in the network. HL neurons can have one or more layers, and the number of neurons in each layer can be one or more. If the initial weight values are all set to 0, in the error backpropagation method, all weight values will be updated the same, and the neural network will not be able to learn normally. For example, in a two-layer neural network, assume that the weights of layer 1 and layer 2 are 0. In this way, when propagating forward, because the weight of the input layer is 0, all the neurons in layer 2 will be passed the same value. All neurons in layer 2 input the same value, which means that all weights in layer 2 will be updated the same during backpropagation. Therefore, the weights are updated to the same value and have symmetric values (duplicate values). This makes the meaning that neural network has many different weights lost. In order to prevent “weight homogenization,” strictly speaking, it is necessary to randomly generate initial values in order to collapse the symmetric structure of weights.

Now, it has been proved theoretically that BPNN with only one HL has the ability to approach any nonlinear continuous function [15]. Therefore, only one layer of HL is generally used when BPNN is used.

In the three-layer BPNN model, general HL neurons and OL neurons use Sigmoid function as the excitation function [16, 17]. There are two forms of Sigmoid functions: Log-Sigmoid function and Tan-Sigmoid function.

The Log-Sigmoid function expression is

(1) $$\begin{array}{c} f\left(x\right)=\frac{1}{1+e^{-x}}. \end{array}$$

The expression of Tan-Sigmoid function is

(2) $$\begin{array}{c} f\left(x\right)=\frac{1-e^{-x}}{1+e^{-x}}, \end{array}$$

where *x* represents the input of the upper neuron, and this function can map the input value to the interval (−1, 1).

The application process of the BPNN model mainly includes two processes:

1. Calculate that output vector according to the forward propagation of the input vector;
2. According to the error between the output vector and the expected vector, the weights and thresholds between IL and HL and between HL and OL are reversely updated.

The standard BPNN algorithm uses the method of gradient descent of error function to learn until the sum of error squares between the actual output of the model and the expected output of the model is the smallest.

Figure 2 is the flow chart of the BPNN structure.

BPNN model is one of the most widely used neural network models so far. It has the characteristics of good nonlinear mapping ability, distributed information storage, self-learning and adaptive ability, parallelism, and strong robustness.

The BP neural network is trained to model the model, and then the output value of the model is calculated according to the input data of the training set. Then, compare the model output with the actual output to update the weight and width of the neural network in reverse until the network model reaches a relatively stable state [18].

BPNN model can work normally even if the external information is partially lost or the network is partially damaged, and it will not have much influence on the training results, so BPNN has strong robustness.

### 3.2. Optimization of Customs Clearance Efficiency between Guangdong and Hong Kong

#### 3.2.1. Factors Affecting Customs Clearance Efficiency

Customs clearance is a complex systematic project, involving customs and other related departments such as commodity inspection, frontier defense, and different business departments within the customs. It is not just a matter of one customs clearance business department. As far as the customs is concerned, customs clearance needs the cooperation of other departments including the customs clearance department. This phenomenon reduces the overall efficiency of customs clearance and hinders the improvement of customs clearance efficiency.

Because of the complexity and urgency of the project, the carrier must be professional and efficient personnel, so most employees must receive vocational training. However, due to the particularity of land transportation, it is difficult to attract the company's attention when the operating profit rate is low. Therefore, international logistics companies tend to regard this transportation business as a small part of their business. There are differences in customs, laws, and rules and regulations between Guangdong and Hong Kong. Therefore, the relevant staff are specious about the delivery problems between the two places, lacking proper training links, and eager to set up employees to work, which leads to frequent mistakes, resulting in increased errors in the customs clearance process caused by personnel knowledge problems, which leads to increased costs and customer complaints, leading to a vicious circle.

Customs clearance for land transportation between Guangdong and Hong Kong is usually completed by logistics companies. In order to realize the normal traffic between Guangdong and Hong Kong and complete the distribution work, the license plates of Guangdong and Hong Kong must be equipped. Therefore, if the consignor's delivery location has fixed requirements for vehicles, it should inform the logistics company in advance; otherwise, it will lead to the transportation time exceeding the limit, and even the consignor of export enterprises will pay extra fees. At present, the information of export commodities provided by export enterprises in Guangdong-Hong Kong land transportation customs clearance is incomplete, which affects the speed of customs clearance. Finally, export enterprises need to make up commodity information or other formalities to successfully pass the customs clearance. There is less communication between the two parties, longer waiting time for transport vehicles, higher distribution cost, and lower distribution efficiency.

#### 3.2.2. Construction of Main Process Model of Port Customs Clearance

The particularity of customs is that it has the dual attributes of “law enforcement” and “service.” In order to ensure supervision, many processes cannot be changed, there are historical reasons, and it is also necessary to avoid the risk of clean law enforcement.

At present, according to the actual risk level and classified customs clearance of Guangdong-Hong Kong land transportation, the schematic diagram of the main process model of port customs clearance is shown in Figure 3. The electronic examination documents are divided into three risk levels, and goods go through different customs clearance channels according to the risk levels.

In order to ensure the feasibility of the optimized scheme, the efficiency of the customs clearance “assembly line” will be improved to the maximum extent on the premise of minimum changes to the customs clearance process according to the actual situation. Further refine commodity risk classification and strengthen channel identification. Improve the effectiveness of audit and reduce the waste of time and resources caused by repeated audit. By giving priority to risk assessment and risk classification as much as possible, and adopting more thorough risk classification and customs clearance, we can achieve the purpose of treating different types of goods differently.

If the instructions received in the next link are earlier, the next link can start earlier so that the links can be more closely linked and the flexibility can be improved. When a new process is added to the model, experiments and measurements can be carried out by computer, thus providing a certain basis for model evaluation, optimization, and decision-making.

According to the above-mentioned basic ideas, this paper gives an optimized and improved model for the customs clearance process of Guangdong-Hong Kong land transportation. The original three-level risk level is subdivided into eight-level risks, and the original four-level channels are expanded into eight-level channels. Some links are split and put into different channels according to the characteristics of different channels. The optimization model of the main process of port customs clearance is established as shown in Figure 4.

#### 3.2.3. Application of BP Neural Network Algorithm in Optimization of Customs Clearance Efficiency of Guangdong-Hong Kong Land Transportation

In the feedback neural network, the information in neurons needs to be transmitted forward and backward. Feedback neural network is a dynamic network. Only when the stable condition is satisfied can the network reach a stable state after working for a period of time.

Now, it has been proved theoretically that the BP neural network with only one HL has the ability to approach any nonlinear continuous function [19, 20]. Therefore, in order to reduce the complexity of the BP neural network model, only 3 layers of HL neurons are used in this study. The empirical formula for determining the number of HL neurons is as follows:

(3) $$\begin{array}{c} p=\sqrt{d+m}+\varepsilon ;\;0\leq \varepsilon \leq 10. \end{array}$$

In the formula, *d* is the number of input neurons and *m* is the number of output neurons. According to the above formula and the determined number of input neurons and output neurons, it is known that the number of HL neurons should be between [5, 15].

The neural network model was trained 10 times when HL neurons were 5, 8, 10, and 15, respectively. The data of convergence time, sum of error squares, and so on are shown in Table 1:

According to the experimental data in Table 1, considering the convergence speed of the neural network and training error, the optimal number of HL neurons is 8.

BPNN algorithm has some disadvantages, such as easily falling into local minima in sample training and slow convergence speed in network training. Therefore, in this experiment, when using the BPNN algorithm, the additional momentum method and learning rate adaptive method are used to adjust the learning rate to improve the algorithm.

The additional momentum method can effectively avoid falling into the local minimum during the training of the neural network algorithm. Using the additional momentum method, the change formula of weight and threshold is as follows:

(4) $$\begin{array}{c} \Delta v_{kj}^{\text{new}}=\alpha v_{kj}^{\text{old}}-\eta \frac{\partial E}{\partial v_{kj}},\\ \Delta v_{k0}^{\text{new}}=\alpha v_{k0}^{\text{old}}-\eta \frac{\partial E}{\partial v_{k0}},\\ \Delta w_{ji}^{\text{new}}=\alpha w_{ji}^{\text{old}}-\eta \frac{\partial E}{\partial w_{ji}},\\ \Delta w_{j0}^{\text{new}}=\alpha w_{j0}^{\text{old}}-\eta \frac{\partial E}{\partial w_{j0}}. \end{array}$$

*v*_*k*0_ represents the width of the *k* th output neuron; *w*_*ji*_ represents the weight of the *j* neuron of IL to the I neuron of HL; *w*_*j*0_ represents the width of the *j* neuron of HL. *α* represents momentum factor, and its value is between (0, 1); *η* is the learning rate, its value is between (0, 1), and *E* is the sum of squares of training errors.

After adopting the additional momentum method, if the network training reaches the local minimum, the network model will continue to search for the minimum due to the influence of additional momentum, so it is possible to jump out of the local minimum until the global minimum is found.

The number of input variables of BPNN depends on the complexity of the controlled system. Because the output cannot be negative, the activation function of OL is a nonnegative Sigmoid function, and HL is a positive and negative symmetric Sigmoid function. Therefore, we construct a three-layer BP network with a structure of 4-8-3, and the designed three-layer BPNN structure is shown in Figure 5:

The input and output of the network are

(5) $$\begin{array}{c} O_{j}^{\left(1\right)}=x_{j}j\\ =1∼4. \end{array}$$

The input and output of network HL are

(6) $$\begin{array}{c} {\text{net}}_{i}^{\left(2\right)}\left(k\right)=\sum_{j=0}^{M}w_{ij}^{\left(2\right)}O_{j}^{\left(1\right)},\\ O_{i}^{\left(2\right)}=\left(k\right)=f\left({\text{net}}_{i}^{\left(2\right)}\left(k\right)\right),\;i=1,2,\ldots 8, \end{array}$$

where *w*_*ij*_^(2)^ is the HL weighting coefficient. The upper horns (1), (2), and (3) represent IL, HL, and OL, respectively.

The input and output of the network are

(7) $$\begin{array}{c} {\text{net}}_{l}^{\left(3\right)}\left(k\right)=\sum_{i=0}^{Q}w_{li}^{\left(3\right)}O_{i}^{\left(2\right)}\left(k\right),\\ O_{l}^{\left(3\right)}\left(k\right)=g\left({\text{net}}_{l}^{\left(3\right)}\left(k\right)\right)\;l=1,2,3,\\ O_{1}^{\left(3\right)}\left(k\right)=K_{p},\\ O_{2}^{\left(3\right)}\left(k\right)=K_{i},\\ O_{3}^{\left(3\right)}\left(k\right)=K_{d}, \end{array}$$

where the OL output nodes correspond to three adjustable parameters *K*_*p*_, *K*_*i*_, *K*_*d*_, respectively.

Take the performance index function as

(8) $$\begin{array}{c} E\left(k\right)=\frac{1}{2}{\left(r\left(k\right)-y\left(k\right)\right)}^{2}. \end{array}$$

Generally, the weight coefficient of the network is modified according to the gradient descent method [26], that is, the negative gradient direction of the weight coefficient is searched and adjusted according to *E*(*k*) [21, 22].

## 4. Result Analysis

Support vector machine SVM is an important machine learning algorithm. Here, MATLAB software is used to design an SMO algorithm to achieve optimal classification. There are 30 input neurons, 3 output neurons, 8 HL neurons, and only one layer of HL neurons. Establish the algorithm model and predict the customs clearance within a week, as shown in Table 2.

The quadratic exponential smoothing method, SVM (Support Vector Machine) model, and neural network algorithm are used to predict the customs clearance volume within a week. The average relative error rate of prediction is shown in Figure 6.

These three forecasting algorithms can predict the next stage of customs clearance to a certain extent. However, sometimes the quadratic exponential smoothing method is the best, sometimes the SVM model is the best, and sometimes the BPNN model is the best, and no algorithm can completely surpass the prediction results of other algorithms. But generally speaking, BPNN is higher than the other two prediction algorithms in the overall prediction level.

When the quadratic exponential smoothing method is used for prediction, the predicted value can only change along one trend. However, when BPNN is used for forecasting, it can reflect various trends of the predicted value in a certain period of time. Compared with these three prediction algorithms, the time spent by the neural network model is much longer than that of the other two algorithms. From the development trend of prediction results, BPNN can predict the development trend of data more accurately than other algorithms.

The PID control of BPNN is used in the closed-loop system, and the closed-loop control system is modeled by SIMULINK in MATLAB. The closed-loop step response curves of the first-order and second-order systems are obtained respectively as shown in Figures 7 and 8.

From the simulation results, it can be seen that none of the algorithms in this paper produce overshoot, which is determined by the improved conjugate gradient method to globally optimize the objective function, thus avoiding the local minimum. Comparing the two simulation results, for the first-order system, the algorithm in this paper has no overshoot while the overshoot of the latter is 7%. For the second-order system, this algorithm has no overshoot while the overshoot of the latter is 19%.

It can be seen that the algorithm in this paper can improve the convergence speed without increasing the complexity of the algorithm and can reach the global optimum or global extreme point along the conjugate direction. Moreover, it does not need to establish an accurate mathematical model of the controlled object, it realizes online tuning of control parameters, and it has strong self-adaptive and self-learning ability.

Customs clearance generally includes four links, namely, declaration, inspection, taxation, and goods release. Then, in a goods customs clearance system, the indicators of customs declaration that we care about are the probability that the customs declaration is immediately satisfied, which is called the satisfaction rate of customs declaration; the percentage of accepted customs declaration forms in all customs declarations that arrive is called service level; and how long can an accepted customs declaration be honored, which is called the waiting time of customs declaration.

For simplicity, we use cost to analyze risk here. The lower the cost, the lower the risk. Take the cost *c*_*i*_ = 2 of a single link and compare the total cost *C* = 10,20,30,40. Using the upper bound approximation and the lower bound approximation, the optimization results of the optimal mechanism setting level are given (see Table 3).

It can be seen from the table that under the premise of the same average completion time, the larger the variance of completion time, the higher the average number of customs declaration in arrears in the system.

The summary of simulation results is shown in Figure 9.

In the optimized BPNN algorithm of Guangdong-Hong Kong customs clearance process based on business priority scheduling, the customs clearance cycle time of the three priority businesses is greatly shortened, the service efficiency is greatly improved, and the working pressure of customs personnel is also reduced, among which the customs clearance cycle time of the highest priority business is shortened most obviously, and it takes only 8.03 h hours on average to complete the whole customs clearance process.

Modern logistics development needs the integration and optimization of resources among enterprises, especially the integration and optimization of logistics resources. Strengthening cooperation among enterprises can avoid vicious competition and improve the utilization rate of resources. In the process of customs clearance by land transportation between Guangdong and Hong Kong, freight forwarding companies should appropriately relax the confidentiality of customer information and disclose the information of vehicles and drivers to customers in time so that customers can know the latest logistics progress. The Hong Kong car transport company should also abide by the industry rules, avoid the phenomenon of “poaching,” and maintain a good long-term cooperative relationship with freight forwarding companies so as to realize the efficient and low-cost operation of land transportation between Guangdong and Hong Kong, and the enterprises in the whole link can achieve a win-win situation.

## 5. Empirical Test and Evaluation of Innovation Ability of Guangzhou Port Logistics Industry Cluster

The index data of Guangzhou is used as the training sample of the BP neural network. According to the evaluation index system of innovation capability of the port logistics industry cluster, three innovation resource input indexes with the largest weight (R&D fund input, national and local innovation technology center input, and patent input) are selected as the input layer of BP neural network model. Two output indicators of innovation resources with the largest weight (port cargo throughput and port total import and export) are selected as output layer neurons of BP neural network model.

Construct BP neural network structure: the number of neurons in the input layer is 3, the number of neurons in the hidden layer is 3 : 7 : 2, and the number of neurons in the output layer is 2. The hidden layer adopts S-type transfer function Tansig, and the transfer function in the output layer is purelin. The BP neural network is trained by the gradient descent method. When the mean square error reaches 0.65 × At 10 : 00, the training ends. Using the sample data, the trained BP network is simulated, and the learning and comparative test results of the network output value and the actual value are obtained.

The BP neural network model was tested 100 times by using the evaluation index data of the innovation ability of the Guangzhou port logistics industry cluster in 2012. It is found that the data errors between the two outputs of the trained BP neural network model and the average value of 100 tests are 099% and 3.20%, respectively, both below 5%. The training effect of the BP neural network is ideal. Secondly, BP neural network is used to evaluate the innovation ability of port logistics industry clusters in Shanghai, Shenzhen, Tianjin, and Xiamen. According to the evaluation results of the BP neural network, the gap between its innovation ability and the Guangzhou port logistics industry cluster is compared.

The results show that the application of the BP neural network algorithm, combined with the port logistics industry cluster innovation ability evaluation system, can better evaluate and analyze the port logistics industry cluster innovation ability quantitatively. The evaluation results can effectively explain the innovation ability level of the urban port logistics industry cluster and guide the city to strengthen the construction and improvement of the innovation ability of the port logistics industry cluster.

## 6. Conclusion

The efficiency of cargo clearance is the key factor restricting the development of land transportation between Guangdong and Hong Kong. However, the Chinese customs has carried out a series of reforms to improve the efficiency of cargo clearance. Taking Guangdong and Hong Kong Customs as examples, this paper establishes the BPNN algorithm and simulates the model. Finally, the simulation results show that the algorithm improves the convergence speed without increasing the complexity of the algorithm, and there is no need to establish an accurate mathematical model of the controlled object, nor to realize the online tuning of control parameters. It can approach nonlinear objects well and has strong adaptability, self-learning ability, and robustness. The customs clearance process after the reform has a shorter cycle and higher customs clearance efficiency. However, due to the lack of systematic analysis of the factors affecting customs clearance efficiency and the lack of corresponding quantitative optimization models to support the establishment of customs agencies, this paper needs further elaboration and analysis in future research.

## Figures and Tables

**Figure 1:** BPNN structure diagram.

**Figure 2:** BPNN structure flow.

**Figure 3:** Main process of port customs clearance before optimization.

**Figure 4:** Optimized main process of port customs clearance.

**Figure 5:** Three-layer BPNN structure diagram.

**Figure 6:** Comparison of experimental results error.

**Figure 7:** Closed-loop step response of first-order system.

**Figure 8:** Closed-loop step response of second-order system.

**Figure 9:** Length of customs clearance period before and after optimization.

**Table 1:** Convergence rate comparison.

Number of HL neurons	The fastest convergence speed (seconds)	Slowest convergence rate (seconds)	Average convergence rate (seconds)	Error sum of squares
5	116	239	177	11.21
8	122	224	182	11.33
10	113	233	199	11.27
15	135	249	208	11.06

**Table 2:** Comparison between output and actual output.

Time	Actual value	Predicted value	Relative error rate (%)
Monday	663	659	0.6
Tuesday	417	404	3.1
Wednesday	825	812	1.6
Thursday	913	896	1.9
Friday	1258	1243	1.2
Saturday	1412	1401	0.8
Sunday	1877	1861	0.9

**Table 3:** Optimization numerical results of optimal mechanism setting level problem.

Quality of service	Optimal service capacity	Optimal cost	Customs declaration satisfaction rate			
			Index	Erlang	Well-distributed	Fixed length
0.71	6	18.32	0.821	0.824	0.847	0.866
0.77	8	47.71	0.836	0.833	0.855	0.871
0.83	8	50.21	0.901	0.847	0.869	0.892
0.91	7	61.21	0.922	0.901	0.889	0.904
0.90	9	66.98	0.968	0.928	0.904	0.923

## Data Availability

The data used to support the findings of this study are available from the corresponding author upon request.
